This article has been retracted.

# Nuclear Matrix Protein 22 in Voided Urine Cytology Efficacy in Risk Stratification for Carcinoma of Bladder

**DOI:** 10.4021/wjon677w

**Published:** 2013-07-15

**Authors:** Monica Sankhwar, Rajender Singh, Satya Narayan Sankhwar, Madhu Mati Goel, Amita Jain, Pushp Lata Sankhwar

**Affiliations:** a Department of Urology King George Medical University, Lucknow, India; b Department of Division of Endocrinology, Central Drug Research Institute (Council of Scientific and Industrial Research), Chattar Manzil Palace Lucknow, India; c Department of Pathology, King George Medical University Lucknow, India; d Department of Microbiology, King George Medical University, Lucknow, India; e Department of Obstetrics and Gynaecology, King George Medical University, Lucknow, India

**Keywords:** Bladder cancer, NMP22, Urine cytology, Cystoscopy, Hematuria

## Abstract

**Background:**

To investigate the nuclear matrix protein NMP22 in voided urine for detection of malignancy in patients with risk factors of symptoms of bladder cancer.

**Methods:**

January 2009 to December 2012, participants included 1,331 patients at elevated risk for bladder cancer due to factors such as history of smoking or symptoms including hematuria and dysuria, patients at risk for malignancy of the urinary tract provided a voided urine sample for analysis of NMP22 protein and cytology prior to cystoscopy. The diagnosis of bladder cancer, based on cystoscopy with biopsy, was accepted as the reference standard. The performance of the NMP22 test was compared with voided urine cytology as an aid to cancer detection. Testing for the NMP22 tumor marker was conducted in a blinded manner.

**Results:**

Bladder cancer was diagnosed in 79 patients. The NMP22 assay was positive in 44 of 79 patients with cancer (sensitivity, 55.7%, 95% confidence interval (CI), 44.1-66.7%), whereas cytology test results were positive in 12 of 76 patients (sensitivity, 15.8%; 95% CI, 7.6-24.0%). The specificity of the NMP22 assay was 85.7% (95% CI, 83.8-87.6%) compared with 99.2% (95% CI, 98 initial endoscopy, including 3 that were muscle invasive and 1 carcinoma in situ.

**Conclusion:**

The noninvasive point-of-care assay for elevated urinary NMP22 protein can increase the accuracy of cytoscopy, with test results available during the patient visit.

## Introduction

Carcinoma of the urinary bladder, the fourth most common cancer in men and the ninth most common cancer in women, results in significant morbidity and mortality. Most patients with bladder cancer receive the diagnosis after they present with gross or microscopic hematuria. At initial diagnosis, approximately 70% of patients have bladder cancers that are confined to the epithelium or sub-epithelial connective tissue [1]. Cigarette smoking is an established cause of bladder cancer, accounting for approximately 50% of the disease burden in the United States and other Western countries [2]. The incidence of bladder cancer is higher in men, individuals older than 60 years, and those exposed to carcinogens in their occupation or environment. Cigarette smoking is the most common risk factor and doubles the risk of bladder cancer, accounting for approximately 50% of the bladder cancer deaths in men and 30% in women [2]. Hematuria and irritative voiding symptoms are the most common symptoms among patients with urinary tract malignancy. Hematuria in bladder cancer can be intermittent, and its degree does not correlate with the severity of underlying disease [3].

A combination of methods is used to evaluate patients at risk for bladder cancer because no single procedure is 100% sensitive. Flexible cystoscopy is an excellent to because it is low risk and generally can be done in the physician’s office under local anesthesia. However, accuracy can be reduced by poor visualization caused by inflammatory conditions or bleeding, and flat urothelial lesions such as severe dysplasia and carcinoma in situ may be difficult to distinguish from normal bladder tissue [4, 5]. For this reason, voided urine cytology is frequently used as an adjunctive noninvasive test, but it is expensive, subjective, and has low sensitivity.

We investigated whether a new, noninvasive urine-based test for the nuclear matrix, protein NMP22 proteomic marker, using monoclonal antibodies in a point of care format, has clinical utility as an aid in diagnosis of bladder cancer and compared its ability to detect cancer with that of voided urine cytology.

## Methods

Patients with cancers other than of the bladder provided a urine specimen for NMP22 protein analysis during a routine visit and did not have endoscopy or voided cytology evaluations. Each patient evaluated for bladder cancer provided a voided urine sample before undergoing cytoscopy. One protein of each sample was sent for routine cytological examinations, either within the institution or at a reference laboratory, according to the standard practice at each participating facility. An aliquot of the remaining specimen was tested for the presence of NMP22 protein by a member of the clinic staff. Each device was identified by study identification number so that the physicians who performed the subsequent cystoscopy were blinded to the NMP22 test results, and the staff members who performed the NMP22 assay were blinded to cystoscopy test results. Technicians who conducted the cytological examinations were physically distant from both the cystoscopy and NMP22 evaluation, and laboratory reports arrived after the cystoscopies had been completed and documented.

### NMP22 assay

Staff members at each office performed the NMP22 assay per protocol by adding 4 drops of voided urine to the sample well of the point of care device. Positive or negative results were read 30 to 50 minutes later in the test window. A built-in control indicated that the assay was complete. There were no other procedural steps.

The IMMP22 point of care device (NMP22 flow immunochromatographic qualitative assay. It detects elevated amount of the nuclear mutotin apparatus protein, which is a abundant component of the nuclear matrix proteins make up the internal structural framework of the nucleus [6, 7] and are associated with such functions as DIMA replication and RNA synthesis [8, 9], as well as regulation and coordination of gene expression [10-12], in tumor cells, nuclear mitotic apparatus protein, which is present in the inter phase nuclear and associated with the organization of mitotic spindles during cell division [13], is elevated concordant with structural/morphological changes characteristic of malignant cell nuclei. Nuclear matrix protein expression varies with cell type of origin [14, 15]. In individuals with bladder cancer nuclear mitotic apparatus protein is released into the urine during cell death. Unlike cytological examination its detection is not dependent on recovery of intact cells. A microtiter plate immunoassay was developed for this protein previously [16].

Two different monoclonal antibodies are used in the NMP22 point of care assay, one as a capture antibody, and one as a reporter. To perform the test, fresh unprocessed urine is added to the sample well of the device and allowed to react with the colloidal gold-conjugated reported antibody. If NMP22 protein is present in the urine, it will interact with the reporter conjugate to form an immune complex. The reaction mixture flows through the membrane, which contains zones of immobilized antibodies. In the test zone, antigen-conjugate complexes are trapped by the capture antibody, forming a visible line if the concentration of NMP22 protein in the urine is a greater than 10 U/mL. A procedural control zone contains an immobilized IgG-specific antibody that will capture the conjugated antibody independently in the presence or absence of the antigen, thereby always producing a visible control line in the window to demonstrate that each device is working properly [17, 18].

### Diagnostic criteria

All patients with risk factors or symptoms of bladder cancer underwent cystoscopy. They were considered positive for malignancy if 1 or more tumors were observed during initial cystoscopy or within the subsequent 3 months. Nine patients with no malignancy found during their initial cystoscopy had a subsequent endoscopy due to continued suspicion, such as increased symptoms. Removed tumors were defined as malignant based on pathological examination. Tumors that were seen endoscopically but not removed were considered positive for malignancy and designated stage (TX) and grade (GX). Reasons that neoplasia were not removed included concurrent health problems that made patients poor candidates for surgery and advanced age. Patients were considered negative for cancer if no tumor(s) was seen endoscopically, or if tissue was biopsied and defined as nonmalignant on the basis of histopathological examination [19, 20].

### Statistical analysis

Sensitivity of the NMP22 test to detect the presence of bladder with true-positive test results (positive NMP22 test result and tumor) divided by the total number of patients with malignancy, as detected by endoscopy. Specificity was defined as the percentage of patients with a negative NMP22 test result who were not diagnosed with tumors. Corresponding 95% confidence intervals (CIs) were calculated for both sensitivity and specificity were calculated for comparison. A positive cytology test result was defined as one in which malignant or dysplastic cells were present.

## Result

### Characteristics of the patients

Demographic and baseline characteristics of the individuals with risk factors or symptoms of bladder cancer are summarized in Table 1.

**Table 1:** Patient’s Demographics and Baseline Characteristics

Variables	No urinary tract disease (n = 567)	Benign disease (n = 685)	Urinary tract cancer (n = 79)	Overall (n = 1,331)
Mean (SD)	54.1 (13.8)	61.7 (13.7)	65.8 (13.3)	58.7 (14.3)
Range	18 - 91	27 - 96	21 - 86	18 - 96
No. (%) of patients				
< 40	90 (15.9)	50 (7.3)	4 (5.1)	144 (10.8)
41 - 50	153 (27.0)	95 (13.9)	5 (6.3)	253 (19.0)
51 - 60	146 (25.8)	171 (25.0)	14 (17.7)	331 (24.9)
61 - 70	94 (16.6)	167 (24.4)	23 (29.1)	284 (21.3)
71 - 80	73 (12.9)	153 (22.3)	26 (32.9)	252 (18.9)
> 81	11 (1.9)	49 (7.2)	7 (8.9)	67 (5.0)
Sex, No. (%) of patients				
Male	225 (39.7)	472 (68.9)	62 (78.5)	759 (57.0)
Female	342 (60.3)	213 (31.1)	17 (21.5)	572 (43.0)
Race				
No (%) of patients black, non Hispanic	54 (9.5)	62 (9.1)	4 (5.1)	120 (9.0)
White, non Hispanic	447 (78.8)	572 (83.5)	70 (88.6)	1,089 (81.8)
Hispanic	43 (7.6)	36 (5.3)	5 (6.3)	84 (6.3)
Asia	15 (2.7)	11 (1.6)	0	26 (2.0)
Other	5 (0.9)	1 (0.2)	0	6 (0.5)
Unknown	3 (0.5)	3 (0.4)	0	6 (0.5)

Among the 1,331 patients who had cystoscopies, 79 (6%) and cancer, 685 (51%) were diagnosed with 1 or more benign urological conditions, and 567 (43%) had no cystoscopic evidence or urinary tract disease. The mean age of the patients with bladder tumors was 65.8 years (range, 21 - 86 years), and they comprised 3 times as many mean as women. Staging information was available for the 72 cancers that were surgically removed. The 7 tumors seen during cystoscopy but not excised were categorized as TX. Of the cancers with pathological staging data, 62 were superficial (stages Ta, Tis, or T1), and 10 were muscle invasive (T2-T3). Pathological determination of grade was available for 70 of the 72 removed tumors. Of these, 27 were well differentiated (low grade), 18 were moderately differentiated (medium grade), and 25 were poorly differentiated (high grade). A total of 27 cancers were muscle invasive (T2 or T3) and/or poorly differentiated (high grade). No patients had detectable metastases or involvement of regional lymph nodes. The NMP22 test results were available for all patients with risk factors (1,331), and cytology test results for 1,287 of the patients with risk factors, including 76 of the 79 diagnosed with cancer.

### Detection

Initial cystoscopy alone detected 88.6% (70/79) of the cancers. The remaining 9 malignancies were identified during subsequent cystoscopies conducted due to continued suspicion, such as increased symptoms within 3 months of the initial evaluation. The NMP22 assay was positive in 55.7% (44/79), and cytology test results of malignant or dysplastic cells were found in 15.8% (12/76).

The NMP22 test was significantly more sensitive than voided urine cytology when compared using the McNemar x test (x = 24.6, P < 0.001). This difference remains significant after taking into account the inherent variability among the investigational sites using an adjusted McNemar x test (x = 7.0, P = 0.008). This significant difference is also reflected by the CIs for the sensitivity proportions since they do not overlap, at 55.7% (85% CI, 44.1-66.7%) for the NMP22 test vs 15.8% (95% CI, 7.6-24.0%) for cytology. The positive predictive values of the NMP22 assay and cytology were 19.7% (95% CI, 14.5-25.0%) and 94.9% (95% CI, 93.6-96.1%), respectively (Table 2).

**Table 2:** Sensitivity of NMP22 Assay and Voided Cytology by Stage and Grade of Cancer (n = 72)

	No. with positive test result/total no. with bladder cancer	Sensitivity % (95%Cl)	No. with positive test results/total no. with bladder cancer	Sensitivity % (95%Cl)
Stage				
Ta	14/30	46.7 (28.3 - 65.7)	2/28	7.1 (1.0 - 23.5)
T1	4/5	80.0 (28.4 - 99.5)	3/5	60.0 (14.7 - 94.7)
T2, T2a	6/6	100 (54.1 - 100)	2/6	33.3 (4.3 - 77.7)
TX	4/7	57.1 (18.4 - 90.1)	0/7	0 (0 - 41.0)
Noninvasive: Ta T1	31/62	50.0 (37.0 - 63.0)	10/60	16.7 (8.3 - 28.5)
Muscle invasive: T2-T3	9/10	90.0 (55.5 - 99.8)	2/9	22.2 (2.8 - 60.0)
Grade				
Well differentiated	13/27	48.2 (28.7 - 68.1)	0/25	0 (0 - 13.7)
Moderately differentiated	9/18	50.0 (26.0 - 74.0)	3/18	16.7 (3.6 - 41.4)
Poorly differentiated	18/25	72.0 (50.6 - 87.9)	9/24	37.5 (18.8 - 59.4)
Gx (Grade unknown)	4/9	44.4 (13.7 - 78.8)	0/9	0 (0 - 33.6)

The same methods were used to compare the specificity proportions and demonstrated that cytology was significantly more specific than the proteomic assay (x^2^ = 149.6 P < 0.001), at 99.2% (95% CI, 98.7-99.7%) vs 85.7% (95 CI, 83.8-87.6%), respectively. The difference remains significant after taking variability among the sites into account (adjusted McNemar test x^2^ = 9.0, P = 0.003). The negative predictive values of the IMMP22 assay and cytology were 96.8% (95% CI, 95.6-97.8%) and 94.9% (95% CI, 93.6-96.1%), respectively.

Ten of the 79 malignancies were muscle invasive. Initial cystoscopy visualized 6 (60%) of these, compared with the NMP22 test, which identified 9 (90%) with elevated protein marker. By comparison, voided cytology was positive in only 2 (22%) of the 9 patients with muscle-invasive disease for whom test results were available. The NMP22 assay was also positive for a patient diagnosed with carcinoma in situ after an initial cystoscopic report of benign disease. Thus, a total of 4 potentially life-threatening tumors (T2 G2 of the ureter; T2 G3, Tis G3, and T3 G2 of the bladder) were detected by the NMP22 test but not visualized in the first cystoscopy. Once of the 4 tumor was located in the ureter and therefore outside the viewing area of the cystoscope. Urine tests are often added to an evaluation to identify urinary tract tumors such as this. The combination of the NMP22 test and cystoscopy detected 93.7% of malignancies vs 88.6% for initial cystoscopy alone (P = 0.26). Cytology detected 2 of the 4 cancers not seen in the initial endoscopy, but which were positive by the NMP22 assay. Among the most aggressive malignancies, those that were poorly differentiated (high grade) and/or muscle invasive (stage T2 or T3), the NMP22 test result was positive in 74% (20/27) compared with cytology, which was positive in 39% (10/26). Of the superficial cancers (Ta, Tis, T1) that were moderately or well differentiated (medium of low grade), with 5% (2/41) for cytology. Overall, the point-of-care assay detected 32 malignancies missed by cytology: 11 Ta, 10T1, 4T2, 2 T3, 1 Cis, and 4 TX. Voided cytology was positive in only 2 cancer patients for whom the NMP22 test result was negative, both T1 G3.

The specificity of the NMP22 assay was 90.3% among individuals with symptoms but with no evidence of urinary tract disease seen during cytoscopy, and 85.7% overall (Table 3).

**Table 3:** Specificity of NMP22 Assay

Patients with risk factor for bladder cancer*	No. with negative test result/total no. without bladder cancer	Specificity, % (95% confidence interval)
No urinary tract disease (with risk factor)	512/567	90.3 (87.6 - 92.6)
Benign prostatic hypertrophy/ prostatitis	231/280	82.5 (77.5 - 86.8)
Cystitis/inflammation / trigonitis urinary tract infection	97/125	77.6 (69.3 - 84.6)
Erythema	42/51	82.4 (69.1 - 91.6)
Hyperplasia/ squamous/ netaplasia / cysts and polyps	41/53	77.4 (63.8 - 87.7)
Calculi	29/40	72.5 (56.1 - 85.4)
Trabeculations	175/217	80.7 (74.7 - 85.7)
Other benign disease, kidney and genitourinary	179/220	81.4 (75.6 - 86.3)
Other cancer history, non bladder +	7/8	87.5 (47.3 - 99.7)
Other active cancer, non bladder ++	33/38	86.8 (71.9 - 95.6)

All risk patients in the study were undergoing an evaluation for bladder cancer that included cytoscopy, so false-positive test results did not require any additional procedures. Cytology demonstrated a specificity of 99.2% among patients with symptoms and was not performed for individuals with non-bladder cancer. Of the 39 patients with active cancers other than bladder, the NMP22 assay was negative in 86.8% (33/38) and positive in 13.2% (5/38).

## Discussion

Prognosis and survival of individuals with bladder cancer are related to the stage of the malignancy at the time of detection. Approximately 50% of patients with muscle-invasive disease at first diagnosis demonstrate a recurrence within 2 years of surgery, despite apparently adequate surgical resection. The majority of these patients will experience a cancer-related death within 5 years of diagnosis [21]. By comparison, tumors treated while still confined to the epithelium have lower recurrence rates and progress to higher stages and grades less often, thereby improving patients longterm outcome [22, 23]. In addition, early stage disease can be treated by bladder-sparing thereby rather than cystectomy, the standard for advanced disease, which impacts quality of life as well as survival.

The direct cost of treatment for patients with metastatic genitourinary cancer has been estimated to be more than 6 times greater than for those patients with localized disease for the same period of time [24]. The challenge therefore is to improve detection of bladder cancer without adding increased risk or discomfort to the patient.

Cystoscopy is integral to the diagnosis of bladder cancer, allowing the physician to visualize the bladder wall directly. The sensitivity of cystoscopy is very good, but hematuria and other conditions can obscure lesions, and flat neoplasia can be confused with erythema. As seen in this study, even later-stage cancers are sometimes missed during endoscopy. The precise rate of false-negative during cystoscopy test results is difficult to determine, but estimates range from 10% to 40% [25]. In this study it was 11.4%. For this reason, physicians frequently use multiple tools to aid in diagnosis of bladder cancer, including urinalyses and imaging of the upper tract.

Voided cytology has been a widely accepted adjunctive test to cystoscopy because it is noninvasive. This method involves visual assessment of morphological changes and therefore (low-grade) tumors or both are less likely to exfoliate cells spontaneously because the strong intercellular attachments are better preserved, and the degree of morphological departure from normal is less, making recognition difficult [26-28]. This results in low sensitivity, approximately 15% to 30% in early stage cancers [29, 30]. The high specificity of cytology is offset by low sensitivity, ambiguous test results, expense, and time lag to obtain reports.

We found that the NMP22 test is a useful adjunctive tool in the evaluation of patients at risk for bladder cancer and that it identified several malignancies missed by initial than for cytology (85.7% vs 15.8%), with test results available during the patient visit. The NMP22 protein is the only tumor marker approved by the FDA as an aid in the initial diagnosis of bladder cancer, and the test has been waived under the Clinical Laboratory Improvement Act so it can be performed in any physician’s office. The cost of urine tests varies by location. The average Medicare reimbursement for voided cytology is approximately $56, compared with $24 for the NMP22 point of care assay [31].

Among study patients with the highest risk for bladder cancer, men older than 60 years with a history of smoking, the positive predictive value of the NMP22 test was 37%. This is higher than the 20% to 30% predictive value typically reported for prostate specific antigen in men who have an elevated risk of prostate cancer, those with levels between 4 to 10 ng/mL [32-35].

### Conclusion

In conclusion, the NMP22 assay may be useful adjunct to cystoscopy for diagnosing bladder cancer. Studies in different patient populations are necessary to further define the role of this assay in patients with risk factors and symptoms suggestive of possible bladder cancer.
